This article has been retracted.

# A Study on the Impact of Regional Total Factor Production in Digital Economy Based on Fuzzy Hierarchical VISC Algorithm

**DOI:** 10.1155/2022/6903836

**Published:** 2022-02-26

**Authors:** Haixiang Li, Weixian Xue

**Affiliations:** ^1^School of Economics and Management, Xi'an University of Technology, Xi'an 710048, China; ^2^School of Humanities and Management, Xi'an Traffic Engineering Institute, Xi'an 710300, China

## Abstract

The classification inaccuracy occurs to the evaluation calculation of the total factor production impact in the traditional digital economy development area. This paper applies the fuzzy hierarchical (Visualization in Scientific Computing, VISC) algorithm to the calculation method of the total factor production impact evaluation in the digital economy development area. The quantitative recursive method is used to evaluate the ability of the data information model, to achieve the ability of controlling the acquisition of characteristic resources, and complete the classification and summary of the index parameters of the total factor production impact of the digital economy development area. Finally, the experiment proves that this calculation method is used to develop the evaluation of the impact of total factor production digital economy development area and improve the information integration and analysis capabilities, the accuracy of the evaluation of the impact of total factor production, and the efficiency of the use of digital economy development resources.

## 1. Introduction

As an important transportation infrastructure, several regions are also windows for foreign economic development, providing a guarantee for regional economic development and trade. Since the new century, due to the expansion of city scale and the continuous improvement of regional functions, the digital economy development area is not only the main link of economic development, but also a key link in the economic structure. The transformation of the business structure of the digital economy development area has also become an important research topic [1, 2]. Compared with the traditional regional business development model, the all-factor production structure can effectively utilize the resource advantages of the digital economy development area, reduce the risk of operation, and improve the regional profitability. Therefore, it has been widely used in many digital economy development areas. Digital economy development areas are difficult to get rid of traditional thinking patterns when determining all-factor production strategies. In many cases, companies do not fully consider the total factor production strategy, and the effect is usually not significant. For example, the management system is not sound or the industry to be expanded is inappropriate, which may cause the failure of the regional total factor production strategy and will eventually drag down the main production industries in the region. How to choose an appropriate business strategy for a digital economy development area will be a serious test for regional business managers [3].

After the 1990s, digital economy promoted a large number of new industries, new formats, and new models, and the research of digital economy began to sprout. So far, the research on digital economy mainly focuses on the following aspects: first come the definition and evolution characteristics of digital economy [4]. The essence of digital economy is a special economic form of trading goods and services in a virtual way. Its development is closely related to the information and communication technology industry and accelerates the penetration and change of the operation mode of relevant industries. Chinese scholars have been studying and deepening the connotation and characteristics of digital economy since 2008. He Xiaoyin believes that digital economy is not only a trade behavior dominated by e-commerce, but also an economic process of manufacturing and providing digital products and services; Kang Tiexiang uses a nondefinition method to describe in detail the remarkable characteristics of digital economy, such as virtuality, high permeability, and values added; Yang Xinming expounds the digital economy by analyzing the economic logic of digital economy to the transformation of traditional economy. Second, it introduces the development strategy of digital economy at home and abroad [5]. In order to protect the digital content industry, the British government promulgated the digital economy 2010 law in 2010; in order to achieve the objectives of broadband construction, government development, and Internet education, the Australian government launched the national digital economy strategy in 2011. Third, there is the calculation method of digital economy. Kang Tiexiang uses the sum of the total added value of the digital industry sector and the added value created by digital auxiliary activities to calculate the scale of the digital economy.

Some scholars have found that digital economy can promote economic growth, but few explain its correlation with technological innovation. According to the new economic growth theory, innovation is the driving force of technological progress and the source of economic growth. As an important index to measure technological innovation, total factor productivity analyzes the impact of digital economy on total factor productivity, which is of great significance to speed up the development of economy. Quality development has certain reference value [6].

This article carries an in-depth analysis of the advantages and disadvantages of the selection of total factor production strategies in the digital economy development area and at the same time comprehensively considers domestic and foreign policies, industrial structure, finance, ownership of resources, and corporate managers, etc. The effective implementation of the strategy provides theoretical support and practical testing [7].

## 2. Methodology and Algorithm

To correctly evaluate the impact of total factor production in a digital economy development area, first of all, an information sample model that restricts the impact of total factor production needs a digital economy development area to be built. Combined with the fuzzy hierarchical VISC algorithm, statistical analysis of the factor production impact is carried out. The total factor production impact constraint index parameter of the digital economy development area is a set of nonlinear time series. Construct the total factor production impact analysis and evaluation parameter of the digital economy development area [8].

(1) $$\begin{array}{c} x_{n}=x\left(t_{0}+n\Delta t\right)=h\left[z\left(t_{0}+n\Delta t\right)\right]+\omega_{n}. \end{array}$$

In the formula, *ω*_*n*_ is the error measuring function of evaluation. The solution vector of the analysis and evaluation in the total factor production impact of the digital economy development is calculated by the correlation fusion method, and the digital economy development analysis and evaluation is obtained, and the following conditions are met.

(2) $$\begin{array}{c} \Sigma =\text{diag}\left(\delta_{1},\delta_{2},\ldots ,\delta_{r}\right),\;\delta_{i}=\sqrt{\lambda_{i}},\;\forall i\neq j,\\ \overset{L}{\underset{i=1}{\cup }}S_{i}=V-v_{s}. \end{array}$$

Let *x*_*n*+1_=*μx*_*n*_(1 − *x*_*n*_) be the influence of total factor production in a digital economy development area, where (*I*_*i*_)_*i*∈*N*_={*x*_1_, *x*_2_,…, *x*_*m*_}. For the multivariate group, the analysis and evaluation statistical characteristic distribution sequence x(n) of digital economy development category, the data information flow model of the total factor production impact of the digital economy development area is built based on the previous statistical measurement values:

(3) $$\begin{array}{c} c_{1x}\left(\tau \right)=E\left[x\left(n\right)\right]=0,\\ c_{2x}\left(\tau \right)=E\left\{x\left(n\right)x\left(n+\tau \right)\right\}=r\left(\tau \right)\\ c_{kx}\left(\tau_{1},\tau_{2},\ldots ,\tau_{k-1}\right)\equiv 0,k\leq 3. \end{array}$$

When *q* = 2, the total factor production in the digital economy development area affects the classroom assessment teacher's strength level and the digital economy development resource distribution level, to meet the (2 + 1) dimensional continuous functional condition. In other words, the course of the development of the digital economy needs to be analyzed and evaluated.

(4) $$\begin{array}{c} \psi_{x}\left(\omega \right)=\ln\;\Phi_{x}\left(\omega \right)=-\frac{1}{2}\omega^{2}\sigma^{2}. \end{array}$$

Exclusive analysis appraisal data information flow model of digital economic development built provides an accurate data input basis for the analysis and evaluation of the total factor production and constructs a set of scalar sampling sequence components.

The control objective function for constructing the total factor production impact forecast estimation of the digital economy development area is

(5) $$\begin{array}{c} \underset{x_{a,b,d,p}}{\max}\sum_{a\in A}\sum_{b\in B}\sum_{d\in D}\sum_{p\in P}x_{a,b,d,p}V_{p},\\ \text{s.t.}\sum_{a\in A}\sum_{d\in D}\sum_{p\in P}x_{a,b,d,p}R_{p}^{bw}\leq K_{b}^{bw}\left(S\right),\;b\in B. \end{array}$$

The gray model is used to quantitatively and recursively evaluate the level of total factor production impact capacity of digital economy development. Assuming the historical data {*x*_*i*_}_*i*=1_^*N*^ of the distribution of the total factor production impact capacity of the digital economy development, the initial value of the feature is fixed and the budgetary estimate density functional is estimated from the factor production impact prediction of the digital economy development [9].

(6) $$\begin{array}{c} u_{c}\left(t\right)=Kx_{c}\left(t\right). \end{array}$$

The total factor production impact continuous function of the calculation model of forecast estimation system of the digital economy development area is *u* : *I* × *IR*^*d*^⟶*IR*; after k-1 iterations, *k* ≥ 1, the gray-scale sequence of the total factor production impact of the digital economy development area satisfies N(*k*) < L, and the fuzzy hierarchical VISC algorithm is adopted, to obtain the output indicator of analysis evaluation of the impact of the economic production of all factors, which is the K adjacent sample values of the distributed big data information flow:

(7) $$\begin{array}{c} P_{1J}=\sum_{d_{i}=KNN}\text{Sim}\left(x,d_{i}\right)y\left(d_{i},C_{j}\right). \end{array}$$

The method of fusion of big data information is used to construct the total factor production impact and construct the objective function of analyzing and evaluating the interdomain classification of the distributed data information flow. That is, the objective function of a big data cluster is

(8) $$\begin{array}{c} J_{m}\left(U,V\right)=\sum_{k=1}^{n}\sum_{i=1}^{c}\mu_{ik}^{m}{\left(d_{ik}\right)}^{2}. \end{array}$$

The researched digital economy development curriculum is analyzed, to quantitatively analyze and evaluate the exponential correlation distribution sequence {*x*_*n*_}_*n*=1_^*N*^, find an excellent method of K value, and obtain the quantitative recursive feature extraction result of the digital economy development analysis and evaluation:

(9) $$\begin{array}{c} x_{n}=a_{0}+\sum_{i=1}^{M_{AR}}a_{i}x_{n-i}+\sum_{j=0}^{M_{MA}}b_{j}\eta_{n-j}. \end{array}$$

In the formula, *a*_0_ is the sampling range of the evaluation of the impact of total factor production in the initial stage of digital economy development; *x*_*n*−*i*_ is scalar time series; *b*_*j*_ is the vibration attenuation value of the digital economy development arrangement and analysis evaluation.

Relevant data about the development of the digital economy is listed gradually in the classroom. Mainly, time, class, curriculum, classroom, teacher, and other related factors belong to the optimization decision problem of multiple factors. The fuzzy hierarchical VISC algorithm is a constant weighted evaluation, and the constant easily leads to the unfairness of the evaluation. In the course importance assessment, a part of the component must be activated, and that weight increases with the increase of the factor scores. The method of optimizing the weight vector with the state vector of each indicator (*x*_1_, *x*_2_,…, *x*_*m*_)*W*=(*ω*_1_, *ω*_2_,…, *ω*_*m*_) forms the concept of incentive variable weight. The equilibrium function is integrated into variable weights, and the new variable weight formula is obtained:

(10) $$\begin{array}{c} \omega_{i}\left(x_{1},x_{1},\ldots ,x_{m}\right)=\frac{\omega_{1}x_{1}^{a-1}}{\sum_{i=1}^{m}\omega_{i}x_{i}^{a-1}}. \end{array}$$

When *a*>1, *ω*_*i*_(*x*_1_, *x*_2_,…, *x*_*m*_) is the incentive variable weight. During the process of comprehensive evaluation, if an index value is very large, its comprehensive evaluation value will increase rapidly; that is, *x*_*i*_ will increase, and *ω*_*i*_ will become larger [10].

Construct a constraint of the influence of total factor production in the digital economy development area and use the fuzzy hierarchical VISC algorithm to analyze of the influence of the total factor production in the digital economy development area. The least squares problem is to find the consistent estimate of the resource constraint vector *β* of the total factor production in the digital economy development area, so that ‖*Y* − *Xβ*‖ reaches the minimum, where ‖*·*‖ is the F-norm in the European norm, and the entropy feature extraction value of the total factor production impact constraint feature information in the digital economy development area obtained is

(11) $$\begin{array}{c} P_{\text{loss}}=1-\frac{1-p_{0}}{\rho }=\frac{p_{0}+\rho -1}{\rho }=\sum_{n=1}^{N}p_{K,n}. \end{array}$$

Given that *d*_*i*_ is the disturbance feature vector for the analysis and evaluation of the total factor production impact, the estimation formula of the total factor production impact of the digital economy development area is transformed into the least square solution:

(12) $$\begin{array}{c} z\left(t\right)=x\left(t\right)+iy\left(t\right)\\ =a\left(t\right)e^{i\theta \left(t\right)}+n\left(t\right), \end{array}$$

where *x*(*t*) is the real part of the time series for evaluating the distribution of big data; *y*(*t*) is the imaginary part of the total factor production impact constraint index sequence for the digital economy development area.

The surrogate data method is used to randomize the amplitude of the impact of factor production in the development of the digital economy. It is also possible to perturb the empirical distribution data of the functional analysis evaluation of the k-th digital economy development and obtain the k-th subgroup, which represents the utilization rate of the resource distribution of the digital economy.

(13) $$\begin{array}{c} U_{\text{util}}=\gamma \bar{X}. \end{array}$$

Constructing a hierarchical tree, big data analysis methods are used to establish the main component characteristics of the out-of-time analysis evaluation of the total factor production of the digital economy development, and the ambiguous close filling method is used to solve the similarity of the resource distribution of the digital economy.

(14) $$\begin{array}{c} Sim_{1}\left(d_{i},d_{1j}\right)=\frac{\sum_{k=1}^{M}W_{ik}\times W_{1jk}}{\sqrt{\sum_{k=1}^{M}W_{ik}^{2}}\cdot \sqrt{\sum_{k=1}^{M}W_{1jk}^{2}}}, \end{array}$$

where *d*_*i*_ is the prior distribution feature vector of the total factor production impact of the digital economy development area; *d*_1*j*_ is the K-means clustering center vector of the first-level big data.

Combining the fusion method of linear correlation characteristics, the clustering and integration of the index parameters of the total factor production impact assessment of the digital economy development is realized, and the fusion formula of the output digital economy development resource information is as follows.

(15) $$\begin{array}{c} P\left(w|x\right)=P\left(x|w\right)/P\left(x\right). \end{array}$$

If the quantitative recursive feature is (*N*(*i*)mod*L*) < *m*, the probability density feature of total factor production affecting resource distribution is *p*(*i*)=⌊*N*(*i*)/*L*⌋, the big data stream of the digital economy development area total factor production influence X(i) is divided into p(i) submatrices *X*_*ij*_ whose size is *N*_*ij*_ × *m*, and, through index parameter clustering and integration, the corresponding total factor production impact resource allocation plan is compiled. As a result, the optimization of the influence of all-factor production in the digital economy development area has been realized.

## 3. Analysis and Result

### 3.1. Data Sampling Method

As the most important feature of the digital economy, innovation has created a subversive business model on the “cloud network end” platform of the new generation infrastructure. Driven by Internet enterprises, the construction of a large-scale information platform has accelerated the digitization process of other industries and greatly improved the operation efficiency and business coverage radius of enterprises. The new generation infrastructure maximizes the innovation capacity and innovation potential of individual and small enterprises and reduces the information cost paid by the whole country to the greatest extent. The connection of the Internet promotes the vitality of the industry and endows the industrial innovation value. The digital economy presents connection benefits and output, driving economic growth and prosperity. At the same time, the development level of digital technology affects the digital literacy of the whole people. The digital literacy level of individuals and enterprises reflects their adaptability in the digital age. Whether massive digital information can be effectively obtained, transmitted, and utilized is a necessary condition for enterprises and individuals to improve the level of productivity. For a country, the digital literacy of the whole people determines the comprehensive quality of the country, and it is also an important factor for the country to improve innovation and development in the digital age. The drive of digital economy to regional economic growth is based on the following three aspects: first, drive the demand for innovation. Consumers in the Internet era are also data producers. Big data records commodity purchase behavior, choices, and attitudes, explores consumers' hidden needs, and opens up a huge new consumer market by using electronic online retail. Second, drive innovation supply. As emerging production factors, cloud computing and the Internet have reshaped the market production relations, solved the current problems faced by small- and medium-sized enterprises, such as shortage of funds and insufficient supply of labor and talents, and created emerging business systems and business supply models. Third, improve the “global village market.” Digital economy not only upgrades and transforms traditional industries such as manufacturing, agriculture, construction, and industry, but also improves and transforms service industries such as education and medical treatment with high barriers. Digital economy breaks the industrial boundary and forms a new business ecological model of cross-border industrial chain.

### 3.2. Construction of Digital Economy Index of System

Regarding the selection of digital economy indicators, refer to the indicators and measurement methods issued by the State Statistical Bureau, China Academy of Telecommunication Research of MIIT (CAICT), Tencent Research Institute, etc., and follow the high principle of digital economy development, reliability, and accuracy of indicator sources, to determine the following indicators and weights: first, there is digital infrastructure. Digital facilities are the foundation and the technical support for the development of the digital industry. Five data including Internet penetration rate, mobile phone penetration rate, Internet port access, IPv4 number, and the proportion of CN domain names to the total number of domain names are selected to measure this indicator, and the weight of each indicator is set to 20%. Secondly, there is digital ecologicalization [6, 7]. The ability of technological innovation determines the development realm of an enterprise. The high-frequency iterative technological innovation of the digital economy and the cruelly competitive business ecological model are important characteristics of the digital industry ecology. The ICT industry's fixed investment in the total investment ratio of the whole society, the number of unicorn companies, software business revenue, software product revenue, and software integration revenue indicators are selected to measure the degree of digital ecologicalization, and the weight of each indicator is set to 20%. Thirdly, there are digital talents. The digital economy is a knowledge-based and innovative economy. High-quality talents and high-level scientific research capabilities are the infinite driving force for the sustainable development of the digital economy. In this thesis, the number of degrees awarded by the major in ordinary high schools and high schools is used as the basic data for measuring digital talents, and the weight of each index is set to 50%. Fourthly come the industry value lags behind digit. The added value of industry, the added value of the primary industry, and the added value of the tertiary industry are highly integrated with the digital industry in various fields. However, due to the lagging development of the digital economy in this period, these three indicators are selected to reflect the preliminary industrial development data of the digital economy decolonization and expropriation as a factor of the next development period. The weight of each index is equal to the weight of each level index. The weight of each index is set to 33.3%.

### 3.3. Data Sources and Calculation Results

The above indicator data comes from the State Statistical Bureau and the “Statistical Report on China's Internet Development,” etc. The starting year of the software industry statistics is 2011, so the starting year of the data selected here is 2011. According to the data from 2011 to 2020, the software business revenue, software product revenue, system integration revenue, tertiary industry increase, and industrial value-added index are first standardized. All indicators are weighted, and the results of the digital economy index are shown in Table 1.

Measured from the digital economy index of China's 30 provinces from 2011 to 2020, the leading regions of China's digital economy development are mainly located in the Circum-Bohai-Sea, the Yangtze River Delta, and the Pearl River Delta. Judging from the results at the level, Guangdong Province has always occupied the top position. Based on the guidance of excellent digital infrastructure, industrial development, and policy guidance, Guangdong has become a leader. In 2020, Guangdong committed to building and improving big data foundation and social big data public service platform, etc. Beijing, Shanghai, Tianjin, and Zhejiang continue to develop digitally. These provinces are the areas with a high penetration rate of digital life (such as online car reservation, third-party online settlement, bicycle sharing, and making). The hot spots centered on Sichuan, Hubei, Fujian, Shaanxi, and Shandong have huge potential for economic development. With the provincial capital as the center, we will cooperate with neighboring cities to complement each other and form a digital ecological dialogue. In March 2020, China's first national-level big data comprehensive pilot zone was established in Guizhou Province. In October 2020, the Inner Mongolia Autonomous Region approved China's only national big data comprehensive test zone for infrastructure construction plans and development and also approved two span type comprehensive test zones and four regional demonstration comprehensive test zones for the Beijing-Tianjin-Hebei and Pearl River Delta. They are generally “from observation to exploration, from preliminary construction and development, partial integration, key breakthroughs to balanced development, and this road will move forward.” Large and fast-growing provinces will become a new driving force for China's digital economy development from 2020 to 2030.

### 3.4. Empirical Test

The original data of each variable comes from the “China Science and Technology Statistical Yearbook” (2011–2020) and State Statistical Bureau. The very few missing data are supplemented by the average method. RD (registered trademark) and PG (registered trademark) are flattened according to the index based on 2011.For descriptive statistics of variables, please refer to Table 2.

The descriptive statistical results of the main indicators are shown in Table 3 and Figure 1.

### 3.5. Analysis of Basic Estimation Results

First of all, to determine whether the mixed regression model or the fixed model is to exclude the mixed regression model through F check. Second, through Hausman's inspection, the model is determined, and finally it is shown that the choice of fixed-effect model is scientific [11]. Here, the specific estimation results of the fixed-effect model are shown in Table 4. And the coefficients are all significant at the 1% level, which also verifies the assertion that the digital economy proposed in hypothesis 1 directly promotes regional total factor production. From the point of view of the control variables, the government intervention (gov) and the coefficient of openness to the outside world are obviously negative in the impact on the advancement of the industrial structure. This is basically consistent in the existing research, which shows that when the degree of government intervention is high, it will affect the advanced development of the industrial structure. The degree of opening to the outside world restricts the advancement of the industrial structure. This may be related to China's long-term position at the low end of the international division of labor value chain, and most of its exports are labor-intensive products. The coefficient of marketization level (market) is significantly correct showing that the higher the degree of marketization, the more conducive it is to the realization of advanced industrial structure. Among the influencing factors of industrial structure rationalization, the coefficients of government intervention (gov), marketization level (market), and fixed asset investment level (invest) have dropped significantly, which has a significant role in promoting the rationalization of industrial structure.

In order to verify the mechanism of the digital economy on regional total factor production, this paper uses the intermediary effect model, taking human capital and scientific and technological innovation as intermediate variables, respectively, to analyze the influence mechanism of the digital economy on the advancement of the industrial structure and the rationalization of the industrial structure. The specific analysis results are shown in Table 5. Consistently with hypothesis 2, it indicates that the digital economy has an indirect impact on regional total factor production.

It can be seen from Table 5 that taking human capital as a mesomeric variable, the influence coefficient of the digital economy on human capital is positive, with a significant level of 1%, and the development of the digital economy has a positive impact on the improvement of human capital. The regression coefficients of human capital and digital economy for the advancement of the industrial structure are also significantly positive, and the RI regression coefficients for the rationalization of the industrial structure are all significantly negative; the digital economy shows that, by positively affecting human capital, it can indirectly promote the advancement of the industrial structure and the rationalization of the industrial structure. Other factors remain unchanged. Each additional unit of the comprehensive development of the digital economy will directly increase the level of industrial structure by 0.799 units. Meanwhile, the level of human capital will be increased to 2.797 units, which indirectly rises to 0.080 units. The indirect effect accounts for 9.10% of the total effect. In addition, the comprehensive development level of the digital economy is that, for every additional unit, the rationalization of the industrial structure will directly increase to 0.804 units. While increasing the level of human capital, it will promote the rationalization of the industrial structure, indirectly increasing by 0.233 units, with a total effect of 1.027 units. Indirect effects account for 21.71% of all effects.

When considering technological innovation as a mesomeric variable, it can be seen from Table 4 on technological innovation that the regression coefficient is significant at the 1% significance level. The regression coefficients of technological innovation and digital economy to the advancement of the industrial structure are significantly positive. The digital economy shows that, by improving the level of technological innovation, it can indirectly promote the advancement and the rationalization of the industrial structure. Other factors remain unchanged. For each additional unit of the comprehensive development of the digital economy, the advanced industrial structure will directly increase to 0.776 units, and the level of technological innovation will be increased to 0.038 units, resulting in an indirect increase of 0.103 units in the advanced industrial structure. The effect is 0.879 units, and the indirect effect accounts for 11.72% of the total effect. In addition, for every additional unit of the comprehensive, the rationalization of the industrial structure will directly increase to 0.736 units. While the digital economy promotes the improvement of the level of technological innovation, it indirectly promotes the rationalization of the industrial structure by 0.289 units, with a total effect of 1.025 units. The indirect effect accounts for 28.20% of the total effect.

On the whole, when human capital is a mesomeric variable, the ratios of the digital economy on the advancement and rationalization of industrial structure are 1 and 4 : 1; when technological innovation is the intermediary variable, the ratio of the direct effect and the indirect effect of the digital economy on the advancement of the industrial structure and the rationalization of the industrial structure is 8 : 1 and 3 : 1, respectively. Whether it is based on the advancement of the industrial structure or the rationalization of the industrial structure, the direct effect of the digital economy on regional total factor production exceeds that of the digital economy, improving the indirect effect of human capital accumulation and increasing the level of technological innovation on regional total factor production [12, 13]. Therefore, from the analysis of this paper, the influence of digital economy on regional total factor production is mainly direct promotion, supplemented by indirect promotion.

### 3.6. Nonlinear Analysis

In order to investigate the nonlinear relationship between the digital economy and regional total factor production, the panel threshold model is used to test, and the level of numerical economic development is selected as the threshold variable in this paper. First, confirm the existence of the threshold variable. Empirical results are available on request (due to space limitations, no specific results are listed). There are double thresholds for the impact on the rationalization of the industrial structure of the digital economy, and each threshold is significant at a significant level of 1%, which verifies the hypothesis 3 proposed above. Based on this, the model that sets the specific threshold number is regressed, and the specific nonlinear regression results are shown in Table 6.

The reason for this phenomenon may be that if the development level of the digital economy is low, the digital economy will have a greater role in promoting labor productivity and the optimization of the proportion of the three industries to a certain extent. As the development level of the digital economy increases, the industrial proportional relationship is relatively complete, and the increase in labor productivity is slow. The two will not change as much as when the development level of the digital economy is low. Therefore, the role of the digital economy in promoting the advancement of the industrial structure is weakening.

When it is in the range of [0.550, 0.563], the digital economy significantly promotes the rationalization of the industrial structure. When it is greater than 0.563, the digital economy significantly affects the rationalization of the industrial structure. The promotion effect increases from 0.531 to 0.526, showing the increasing tendency of the boundary effect. As a general-purpose technology, digital technology is applied to various subindustries. The nonlinear impact of the digital economy on the rationalization of the industrial structure is due to the above characteristics. In the early stage of the development of the digital economy, the level of development of digital technology is not high, and it is mainly used in life service fields, such as medical care, education, and shopping, and there may be an insignificant phenomenon. With the rapid development of digital technology, the digital economy has gradually been applied to the field of manufacturing, which has a significant positive impact on optimizing the three industrial structures and promoting the rationalization of the industrial structure.

### 3.7. Analysis of Heterogeneity

In order to test whether on regional total factor production, this paper divides 30 provinces into three regions: east, middle, and west according to the traditional division method that is, three subsamples. Analyze the heterogeneous impact of digital economy on regional total factor production, and the regression results are shown in Table 7.

It can be seen from Table 7 that, from the perspective of the three major regions of the east, middle, and west, the digital economy has a significant role in promoting the advancement of the industrial structure and the regression coefficients are all significant at a significant level of 1%. From the perspective of the degree of digital economy's promotion of advanced industrial structure, the impact of the digital economy has regional differences. Specifically, “the central region < western region < eastern region;” in other words, compared with the eastern region, the central and western regions can obtain more dividends. The digital economy and nonlinearity analyzed above are related to the impact of the advancement of the industrial structure. It not only promotes the advancement of the industrial structure, but also effectively narrows the gap between backward and developed regions. The impact of the digital economy on the rationalization of the industrial structure is different from the impact on the advancement of the industrial structure. The impact of the digital economy on the rationalization of the industrial structure in the eastern region is not significant. From the perspective of the central and western regions, the development of the digital economy has a significant role in promoting the rationalization of the industrial structure, and the regression coefficients are all significant at a significant level of 1%. However, the western region can get more dividends from the development of the digital economy. This proves once again that the development of the digital economy can further reduce the differences in the industrial structure between regions and promote the rationalization and development of the regional industrial structure. In view of the existence of the above economic phenomena, this paper believes that the main reasons are as follows: (1) the digital economy in the eastern region has developed rapidly and the level of development is relatively high. The industry tends to be “service-oriented,” and the dividends of the digital economy that affect the production of the entire region may have been released in advance. (2) The internal gap in the development level of the digital economy in the eastern region is significantly larger than that in other regions. The comprehensive development level index at the beginning of the survey was [0.559, 0.710]. Before the final exam, this level index was in the range of [0.582, 0.939]. The development level of the digital economy with too large gap will produce the phenomenon of “overly sparse” and “overdense” elements. Moreover, because it is not conducive to the coordinated development of the industry, the digital economy in the eastern region has an insignificant impact on the rationalization of the industrial structure.

## 4. Discussion

Research on the impact of digital economy on economic growth and the development trend of digital economy will be done in the future. Liu Chunmei et al. studied the development process and economic characteristics of information economy (digital economy) and made an empirical regression on the quality of economic growth. The results show that information economy affects long-term economic growth by affecting the quality of economic growth. It establishes a vector autoregressive model to regress TFP and finds that information factors have a positive role in promoting TFP. The contribution of digital economy to GDP has gradually increased, bringing millions of new jobs. It is the most active field of economic development in recent years. Digital economy uses science and technology to change the current social lifestyle and industrial model and reshape the core competitiveness of the industry. Based on the above literature analysis, the following is found: firstly, scholars have enriched the meaning and characteristics of digital economy from different angles, dimensions, and directions, but it also makes it difficult to construct indicators to measure digital economy. Secondly, most scholars pay attention to the development trend and development strategy of digital economy, but the research on the impact of all-factor production of digital economy is insufficient.

In this paper, the digital economy index has a significant role in promoting technological innovation. The variable coefficients of each digital economy index are positive, indicating that the development of digital economy brings economic progress. From the perspective of interaction term coefficients, some coefficients are significantly nonzero. Therefore, when there are nonlinear interaction terms, the model can more accurately describe the current phenomenon. The negative coefficient indicates that the smaller the number of effective invention patents of Industrial Enterprises above Designated Size, the greater the marginal effect of digital economy on total factor productivity. This shows that the degree of digital technology innovation in China is still at a low level and the current innovative industries prefer nondigital technology, resulting in the phenomenon that the marginal effect of digital technology is negative. In addition, when digital technology is integrated with real industries, there is an uneven penetration of the three industries, resulting in an unbalanced development of technology driven industries. Secondly, the impact of digital economy index on innovation in different regions is different. From the above regression results, the digital economy in the eastern coastal area plays the greatest role in promoting total factor productivity. At present, digital technology is in the early stage of integration with industry, which is manifested in the overheated development of low-end industries and the overvaluation of domestic economics, meal delivery, and other industries in the capital market. In big cities and mega cities, enterprises are facing more complex competitive markets and more serious information asymmetry, which has greatly changed the survival of the fittest mechanism. We need to pay attention not only to quality and price fluctuation, but also to marketing means and methods. The new innovation model makes the current real economy face great pressure, so the government's ability of governing the market needs to be improved.

## 5. Conclusions

In view of the research on the optimization of the total factor production impact assessment model of the digital economy development area, the digital economy development area total factor production impact method is proposed on the fuzzy hierarchical VISC algorithm proposed in this paper. The fuzzy hierarchical VISC algorithm is used to carry out an analysis of the relevant information of the total factor production impact assessment. Experiments have proved that, by using this calculation method to carry out the evaluation of the total factor production impact of the digital economy development area, the information combination analysis ability is high, the accuracy of the total factor production impact capacity evaluation is greatly improved, and the utilization efficiency of the digital economy development resources is improved.

Based on the above analysis, this paper focuses on the development of digital economy and industrial integration. There is an obvious positive correlation between the development of digital economy and regional distribution, and it has brought great demonstration effect and amplification to urban economic development. Therefore, to promote the innovation and Entrepreneurship of regional digital economy, we need not only large enterprises with leading role, but also small enterprises with strong momentum, also in addition to enterprises that dare to reform and innovate to jointly drive the high-quality development of regional economy.

## Figures and Tables

**Figure 1:** Statistical results of main variables.

**Table 1:** Some calculation results of the digital economy index from 2011 to 2020.

	2011	2012	2013	2014	2015	2016	2017	2018	2019	2020
Beijing	45.7	541.1	65.1	72.3	99.8	121	1236.1	133.8	148.5	175
Tianjin	4	4.9	7.1	8.1	12.1	16.1	20.9	25.3	28.1	31.7
Hebei	3.2	4	4.8	7.5	8.8	10.2	10	10.9	13.2	15.5
Shanxi	2	2.3	2.6	2.9	3.6	4	4.3	4.3	5	5.5
Inner Mongolia	2.1	2.3	2.3	2.5	3.3	3.7	3.8	4.1	4.6	5.1
Liaoning	10.9	140.1	21.3	28.2	48.9	70.7	87.1	94.5	103.8	79.8
Jilin	4.5	5.6	6.6	6.9	9.3	10.8	10.8	12.6	14.4	17.3
Heilongjiang	3.7	4.3	4.5	4.9	5.9	6.7	6.7	7.5	8.7	10.7
Shanghai	19.3	205.1	24.8	28.7	47.5	70.1	69.8	79.9	92.6	104
Jiangsu	27.9	353.1	46.9	62.8	94.7	130.6	1537.1	177.1	204	228.8
Zhejiang	14	154.1	19.7	21.8	31.6	46.4	56.7	64.3	86.5	99.6
Anhui	3.1	3.6	4.2	4.3	5.4	6.4	6.6	8	11.2	21.2
Fujian	9.5	10.9	14.5	19.4	29.8	38.9	44.3	52.4	65.7	76.9
Jiangxi	2.8	3.2	3.3	3.4	4.2	4.8	5	5.3	6.9	8
Shandong	12	142.1	18.7	29	45.2	57.5	69.4	89.6	116.8	134.8
Henan	4.4	5.6	6.3	6.6	8.8	10.4	10.7	12.4	16.3	19
Hubei	4.8	5.8	7.7	8	10.8	13.5	23.9	33.8	37.9	46.6
Hunan	5	5.8	7.3	8.4	11.1	12.1	13.2	15.1	17.4	20
Guangdong	45.7	541.1	65.1	72.3	99.8	121	1236.1	133.8	148.5	175
Guangxi	4	4.9	7.1	8.1	12.1	16.1	20.9	25.3	28.1	31.7
Hainan	3.2	4	4.8	7.5	8.8	10.2	10	10.9	13.2	15.5
Chongqing	2	2.3	2.6	2.9	3.6	4	4.3	4.3	5	5.5
Sichuan	2.1	2.3	2.3	2.5	3.3	3.7	3.8	4.1	4.6	5.1
Guizhou	10.9	140.1	21.3	28.2	48.9	70.7	87.1	94.5	103.8	79.8
Yunnan	4.5	5.6	6.6	6.9	9.3	10.8	10.8	12.6	14.4	17.3
Shaanxi	3.7	4.3	4.5	4.9	5.9	6.7	6.7	7.5	8.7	10.7
Gansu	19.3	205.1	24.8	28.7	47.5	70.1	69.8	79.9	92.6	104
Qinghai	27.9	353.1	46.9	62.8	94.7	130.6	1537.1	177.1	204	228.8
Ningxia	14	154.1	19.7	21.8	31.6	46.4	56.7	64.3	86.5	99.6
Xinjiang	3.1	3.6	4.2	4.3	5.4	6.4	6.6	8	11.2	21.2

**Table 2:** Variable measurement indicators, symbols, and descriptive statistics.

Variable interpretation	*TEP*_*it*_ Technological innovation	DE_*it*_ Digital economy development level	RD_*it*_ Innovative R&D investment	*PG*_*it*_ Innovative R&D output	DE_*it*_*∗*RD_*it*_ Digital economy through TFP marginal effect	DE_*it*_*∗*PG_*it*_ Digital economy through TFP marginal effect
Mean	0.9997	25.2978	1.9491	5.5450	53.4603	191.935
Standard deviation	0.07116	40.6859	1.5922	6.9228	117.6017	496.0943
Maximum value	1.3637	227.72	13.609	63.731	1005.6	4100.6
Minimum value	0.6576	0.21	0.105	0.473	0.21	0.1750

**Table 3:** Descriptive statistics of variables.

Variable	Number of observations	Average value	Standard deviation	Minimum	Max
Indh	210	0.600	0.084	0.477	0.877
Indr	210	0.521	0.303	0.027	1.320
Dig	210	0.600	0.070	0.539	0.939
Hum	210	9.267	0.892	7.514	12.681
Innov	210	0.017	0.011	0.005	0.063
Gov	210	0.251	0.103	0.037	0.628
Open	210	0.256	0.275	0.013	1.343
Market	210	0.600	0.134	0.348	0.868
Invest	210	0.827	0.269	0.210	1.480

**Table 4:** Benchmark regression results.

Explanatory variables	Explained variables			
	Indh	Indh	Indr	Indr
Dig	1.016^*∗∗∗*^ (16.35)	0.880^*∗∗∗*^ (11.83)	−1.042^*∗∗∗*^ (−4.70)	−1.027^*∗∗∗*^ (−3.83)
Gov		−0.193^*∗∗∗*^ (−3.87)		−0.536^*∗∗∗*^ (−2.98)
Open		−0.096^*∗∗∗*^ (−3.09)		−0.179 (−1.60)
Market		0.177^*∗∗*^ (2.25)		−0.633^*∗∗*^ (−2.24)
Invest		−0.017 (−1.40)		−0.123^*∗∗∗*^ (−2.76)
Constant term	−0.01 (−0.26)	0.053 (0.90)	1.146^*∗∗∗*^ (8.60)	1.798^*∗∗∗*^ (8.43)
Sample size	210	210	210	210
	0.599	0.653	0.11	0.218
F value	267.33	65.97	22.05	9.78

*Note.* The *t* statistic value of the estimated coefficient is shown in parentheses. ^*∗∗∗*^indicates the significance level of 1%, 5%, and 10%, respectively. The following table is the same.

**Table 5:** Mesomeric effect regression results.

Variable	Explained variable					
	Hum	Indh	Indr	Innov	Indh	Indr
Mesomeric variable	Hum	Hum	Hum	Innov	Innov	Innov
Dig	2.977^*∗∗∗*^	0.799^*∗∗∗*^	−0.804^*∗∗∗*^	0.038^*∗∗∗*^	0.776^*∗∗∗*^	−0.736^*∗∗*^
	(5.35)	(10.14)	(−2.81)	(8.63)	(8.83)	(−2.31)
Hum		0.027^*∗∗∗*^	−0.075^*∗∗*^			
		(2.74)	(−2.07)			
Innov					2.711^*∗∗*^	−7.607^*∗*^
					(2.16)	(−1.67)
Gov	1.206^*∗∗∗*^	−0.226^*∗∗∗*^	−0.446^*∗∗*^	0.008^*∗∗*^	−0.214^*∗∗∗*^	−0.478^*∗∗∗*^
	(3.23)	(−4.47)	(−2.44)	(2.59)	(−4.25)	(−2.62)
Open	−0.330	−0.087^*∗∗∗*^	−0.204^*∗*^	0.005^*∗∗∗*^	−0.109^*∗∗∗*^	−0.141
	(−1.42)	(−2.83)	(−1.82)	(2.68)	(−3.48)	(−1.24)
Market	0.814	0.155^*∗∗*^	−0.572^*∗∗*^	0.006	0.161^*∗∗*^	−0.589^*∗∗*^
	(1.39)	(2.00)	(−2.03)	(1.24)	(2.07)	(−2.09)
Invest	−0.033	−0.017	−0.126^*∗∗∗*^	0.001^*∗*^	−0.021^*∗*^	−0.113^*∗∗*^
	(−0.35)	(−1.35)	(−2.84)	−1.79	(−1.69)	(−2.52)
Constant term	6.801^*∗∗∗*^	−0.131	2.306^*∗∗∗*^	−0.014^*∗∗∗*^	0.091	1.693^*∗∗∗*^
	(15.33)	(−1.47)	(7.13)	(−3.93)	(1.48)	(7.65)
Sample size	210	210	210	210	210	210
*R* ^2^	0.347	0.668	0.237	0.401	0.662	0.231
F value	18.59	58.26	9.02	23.46	56.9	8.70

**Table 6:** Threshold model regression results.

Explanatory variables	Explained variables	
	Indh	Indr
dig(dig<0.777)	1.169^*∗∗∗*^	
	(16.68)	
dig(dig≥0.777)	1.008^*∗∗∗*^	
	(15.83)	
dig(dig<0.550)		−0.136
		(−0.64)
dig(0.550≤dig≤0.563)		−0.351^*∗*^
		(−1.68)
dig(dig>0.563)		−0.526^*∗∗*^
		(−2.60)
Control variable	Control	Control
Sample size	210	210
*R* ^2^	0.761	0.579
F value	92.19	33.93

**Table 7:** Regression results by region.

Explanatory variables	East region		Central region		Western region	
	Indh	Indr	Indh	Indr	Indh	Indr
Gov	0.758^*∗∗∗*^	−0.112	1.487^*∗∗∗*^	−2.114^*∗∗∗*^	1.218^*∗∗∗*^	−6.056^*∗∗∗*^
	(7.49)	(−1.10)	(10.83)	(−4.92)	(6.56)	(−6.85)
Open	−0.481^*∗∗∗*^	−0.378^*∗∗*^	−0.619^*∗∗∗*^	−1.140^*∗∗∗*^	−0.094^*∗*^	−0.268
	(−2.87)	(−2.25)	(−5.83)	(−3.43)	(−1.92)	(−1.16)
Open	−0.136^*∗∗∗*^	−0.009	0.001	1.173^*∗∗∗*^	−0.182^*∗∗*^	0.425
	(−3.26)	(−0.21)	(0.01)	(3.01)	(−2.32)	(1.14)
Market	0.113	0.114	0.123	−0.673^*∗*^	0.160	0.829
	(0.58)	(0.58)	(1.11)	(−1.95)	(1.46)	(1.58)
Invest	−0.006	0.117^*∗∗∗*^	−0.017	−0.142^*∗∗∗*^	−0.014	−0.127^*∗*^
	(−0.22)	(3.97)	(−1.08)	(−2.83)	(−0.89)	(−1.70)
Constant term	0.222	0.236	−0.212^*∗∗∗*^	2.348^*∗∗∗*^	−0.105	3.995^*∗∗∗*^
	(1.36)	(1.44)	(−2.98)	(10.56)	(−1.14)	(9.10)
Sample size	77	77	56	56	77	77
*R* ^2^	0.734	0.290	0.802	0.753	0.597	0.530
F value	33.68	4.98	34.87	26.14	18.04	13.74

## Data Availability

The data used to support the findings of this study are available from the corresponding author upon request.
